# Midkine promoter-based conditionally replicative adenovirus therapy for midkine-expressing human pancreatic cancer

**DOI:** 10.1186/1756-9966-27-30

**Published:** 2008-08-21

**Authors:** Eiji Toyoda, Ryuichiro Doi, Kazuhiro Kami, Tomohiko Mori, Daisuke Ito, Masayuki Koizumi, Atsushi Kida, Kazuyuki Nagai, Tatsuo Ito, Toshihiko Masui, Michihiko Wada, Masatoshi Tagawa, Shinji Uemoto

**Affiliations:** 1 Department of Hepato-Biliary-Pancreatic Surgery and Transplantation, Kyoto University, Japan; 2 Division of Pathology, Chiba Cancer Center Research Institute, Chiba, Japan

## Abstract

**Background:**

To develop a novel therapeutic strategy for human pancreatic cancer using a midkine promoter-based conditionally replicating adenovirus.

**Methods:**

We examined midkine mRNA expression and midkine protein expression by seven human pancreatic cancer cell lines (AsPC-1, BxPC-3, CFPAC-1, HPAC, MIAPaCa-2, PANC-1, and Suit-2), as well as by non-cancerous pancreatic tissue and pancreatic cancers. Midkine promoter activity was measured in cancer cell lines by the dual luciferase reporter assay. Adenoviral transduction efficiency was assessed by fluorescent staining of cancer cell lines using adenovirus type 5 containing the green fluorescent protein gene (Ad5GFP). Replication of adenovirus type 5 containing the 0.6 kb midkne promoter (Ad5MK) was assessed by the detection of E1 protein in cancer cell lines. The cytotoxicity of Ad5MK for cancer cells was evaluated from the extent of growth inhibition after viral infection. Infection and replication were also assessed in nude mice with subcutaneous Suit-2 tumors by intratumoral injection of Ad5MK, Ad5GFP, or vehicle. E1a mRNA expression in the treated tumors and expression of the replication-specific adenoviral hexon protein were evaluated. Finally, the anti-tumor activity of Ad5MK against intraperitoneal xenografts of Suit-2 pancreatic cancer cells was examined after intraperitoneal injection of the virus.

**Results:**

Both midkine mRNA expression and midkine protein expression were strong in AsPC-1 and CFPAC-1 cell liens, moderate in BxPC-3, HPAC, and Suit-2 cell lines, and weak in PANC-1 and MIAPaCa-2 cell lines. Expression of midkine mRNA was significantly stronger in pancreatic cancers than in non-cancerous pancreatic tissues. The relative luciferase activity mediated by the 0.6 kb midkne fragment in AsPC-1, PANC-1, and Suit-2 cell lines was approximately 6 to 20 times greater than that in midkne-negative MIAPaCa-2 cell lines. Pancreatic cancer cell lines exhibited a heterogeneous adenoviral transduction profile. E1A expression was higher in cell lines with strong midkine expression than in cell lines with weak midkine expression. Ad5MK showed much greater cytotoxicity for midkine-expressing Suit-2 and PANC-1 cell lines than for midkine-negative MIAPaCa-2 cell lines. In the Suit-2 subcutaneous xenograft model, expression of E1A was detected in Ad5MK-treated tumors, but not in untreated and Ad5GFP-treated tumors. In the Suit-2 intraperitoneal xenograft model, the Ad5MK group survived for significantly longer than the Ad5GFP, PBS, and untreated groups.

**Conclusion:**

Ad5MK has an anti-tumor effect against human pancreatic cancer cell lines that express midkine mRNA. Midkine promoter-based conditionally replicative adenovirus might be a promising new gene therapy for pancreatic cancer.

## Background

Pancreatic cancer is one of the most lethal malignant tumors, and it was estimated that approximately 200,000 people died of this cancer worldwide in the year 2000 [1]. It is the fifth leading cause of cancer death in Japan and the fourth in the United States [2]. Unfortunately, the pancreas is located at an inaccessible site within the abdomen, making the diagnosis of pancreatic cancer more difficult than that of other digestive tract cancers. Therefore, most patients with pancreatic cancer are diagnosed late after progression of their disease. Furthermore, pancreatic cancer frequently infiltrates neighboring tissues or vessels at an early stage, leading to a poor prognosis.

In the United States, the 1-year and 5-year survival rates of patients with pancreatic cancer are less than 25% and 5%, respectively [3]. At present, surgical resection provides the only chance of cure for these patients, but it has been reported that about 90% of patients do not undergo pancreatic resection and 58% are only given palliative treatment [4]. Moreover, recurrence after surgical resection is very common. We do not have any effective nonsurgical treatments for pancreatic cancer, because it shows strong resistance to the currently available chemotherapy and radiotherapy protocols [5]. In order to improve the clinical outcome, new modalities for the treatment of this disease are required.

Gene therapy using oncolytic viruses is one of the approaches that should be considered. The strategy of this therapy is to exploits the lytic property of virus replication to kill tumor cells. Recent knowledge of molecular biology makes it possible to modify viruses to target specific molecules or signal transduction pathways in cancer cells. Oncolytic viruses which are developed to be able to infect and replicate selectively in malignant tumor cells can spread and destroy malignant tumors without adverse effects in normal tissues.

To achieve tumor-selective viral replication, one approach has been the replacement of endogenous viral sequences with a tissue- or tumor-specific promoter. A number of tumor promoter genes such as α-fetoprotein [6], carcinoembryonic antigen [7], erbB-2 [8]and prostate-specific antigen [9,10] have been used to restrict the expression of suicide genes both *in vitro *and *in vivo*.

Midkine is a heparin-binding growth factor that is induced by retinoic acid in embryonal carcinoma cells, and it may be another candidate for this purpose [11]. The biological roles of midkine are diverse and it is closely linked to neural development [12,13] as well as to the pathogenesis of neurodegenerative diseases. At the same time, midkine is involved in the development of cancer because of its mitogenic effect [14], promotion of angiogenesis [15], anti-apoptotic activity [16], fibrinolytic activity [17], and transforming activity [18].

Midkine expression is increased in a number of malignant tumors, including esophageal, stomach, colon, hepatocellular, breast and pancreatic carcinoma, when compared with the level of expression in adjacent non-cancerous tissues [19-22]. In contrast, the expression of midkine in normal human tissues is quite limited, with moderate expression in the kidneys and weak expression in the lungs, colon, and thyroid gland [19,20,23].

On this basis, the midkine promoter could be a potential candidate for use in suicide gene therapy. Here, we demonstrate that an adenovirus vector encoding the essential adenoviral E1A gene under the control of 0.6 kb midkine promoter showed specific replication in midkine-expressing pancreatic cancer cell lines and not in non-midkine-expressing cells, and that Ad5MK selectively prevented tumor growth both *in vitro *and *in vivo*.

## Methods

### Cell culture and tumor samples

Seven human pancreatic cancer cell lines were used. AsPC-1, BxPC-3, CFPAC-1, HPAC, MIAPaCa-2, and PANC-1 cells were obtained from the American Type Culture Collection (Rockville, MD), and were maintained in the medium recommended by the ATCC at 37°C in a humidified atmosphere of 5% CO_2_. Suit-2 cells were kindly provided by Dr. Tomoda (National Kyushu Cancer Center, Fukuoka, Japan), and were cultured in DMEM (Gibco-BRL, Grand Island, NY) with 10% fetal bovine serum (FBS) (ICN Biomedicals, Aurora, Ohio). Human embryonic kidney (HEK) 293 cells were purchased from RIKEN Bioresourse Center (Tukuba, Ibaragi, Japan). Each culture medium contained 100 units/ml of penicillin and 0.1 mg/ml of streptomycin (Gibco-BRL).

Pancreatic cancer tissues were obtained from 22 patients who underwent pancreatectomy for ductal carcinoma at our Department. Other pancreatic malignancies were excluded, such as intraductal papillary mucinous adenocarcinoma, acinar cell carcinoma, and endocrine tumors. Informed consent was obtained from each patient according to our Institutional guidelines. A resected specimen was immediately examined by inspection and palpitation at the operation room. A part of malignant or normal tissues considered was cut by surgical knife and it was divided two pieces. One for the tissue samples to extract RNA was immediately frozen in liquid nitrogen and stored at -80°C, the other was fixed in 10% formalin solution to make a paraffin block and performed with HE staining to evaluate pathologically.

### Antibodies

Rabbit polyclonal anti-midkine antibody was kindly provided by Dr. Kadomatsu (Nagoya University School of Medicine, Nagoya, Japan). The following antibodies were purchased; mouse monoclonal anti-E1A (Ad2/Ad5) antibody (clone M73 #05-599) from Upstate Biotechnology (Lake Placid, NY), goat anti-mouse IgG (#62-6500) and HRP-goat anti-mouse IgG (#81-6520) from Zymed Laboratories (South San Francisco, CA), and mouse monoclonal anti-β-actin (clone AC-15 #A-5441) from Sigma (St. Louis, MO). Anti-adenoviral hexon protein antibody was included in the Adeno-X rapid titer kit (BD Biosciences Clontech, Palo Alto, CA).

### RNA extraction and reverse transcription-polymerase chain reaction (RT-PCR)

Total cellular RNA was prepared using TRIZOL Reagent (Life Technologies, Rockville, MD) and cDNA was obtained from 1 μg of total RNA by the random primer method with a First-Strand cDNA Synthesis kit (Pharmacia Biotech, North Peapack, NJ) according to the manufacturer's instructions. Five microliters of first-strand cDNA solution was subjected to the polymerase chain reaction (PCR) with synthetic oligonucleotide primers (NIPPON EGT, Toyama, Japan). For RT-PCR analysis of human adenovirus type 5 E1A, a pair of primers (5'-ATGAGACATATTATCTGCCACGG-3'/5'-TAGACAAACATGCCACAGGTCC-3') was used and PCR was done for 35 cycles at 54°C, yielding a product of 551 base pairs. The reproducibility of the technique and quality of the total RNA were confirmed by amplifying β-actin as well (primers: 5'-GGCATCGTGATGGACTCCG-3'/5'-GCTGGAAGGTGGACAGCGA-3'; product: 613 base pairs).

### Quantitative RT-PCR

To assess midkine gene expression, we used quantitative real-time RT-PCR analysis based on the TaqMan fluorescence method, which employs a dual-labeled non-extendable oligonucleotide hydrolysis (TaqMan) probe in addition to the two amplification primers. The probe contains 6-carboxy-fluorescein (FAM) as a fluorescent reporter dye, and 6-carboxytetramethyl-rhodamine (TAMRA) as a quencher for its emission spectrum. During the extension phase of PCR, the probe hybridizes to the target sequence and is then cleaved by the 5' to 3' exonuclease activity of Taq polymerase. The increase in the fluorescence of the reporter is proportional to the amount of specific PCR products, providing highly accurate and reproducible quantification. The level of reporter dye fluorescence is assessed with an automated sequence detector combined with analysis software (ABI Prizm 7700 Sequence Detection System; PE Applied Biosystems, Foster City, CA). Reaction conditions were set according to the manufacturer's protocol. The following primers and TaqMan probe were used for analysis. The midkine-specific primers were 5'-CGACTGCAAGTACAAGTTTGAGAAC-3' (upstream primer) and 5'-TCTCCTGGCACTGAGCATTG-3' (downstream primer), while 5' (FAM)-AAGGCACCCTGAAGAAGGCGCG-(TAMRA) 3' was the TaqMan probe.

The PCR parameters were 95°C for 10 min (for activation of Taq-Polymerase), followed by 40 cycles of 95°C for 15 s and 60°C for 1 min. Amplification of β-actin for quality control and normalization was done with the TaqMan β-actin Control Reagent kit (PE Applied Biosystems), which utilizes standard TaqMan probe chemistry.

### Western blot analysis

Cells were lysed in RIPA buffer containing 50 mM HEPES (pH 7.0), 250 mM NaCl, 0.1% Nonidet P-40, 1 mM phenylmethylsulfonylfluoride (PMSF), and 20 μg/ml gabexate mesilate, and were incubated on ice for 10 minutes. Then the lysate was sonicated for 10 sec. Total extracts were cleaned by centrifugation at 15,000 rpm for 10 min at 4°C and the supernatants were collected. The protein concentration was measured with the BCA protein assay reagent (Pierce, Rockford, IL). Lysates were resuspended in one volume of gel loading buffer, which contained 50 mM Tris-Hcl (pH 6.7), 4% SDS, 0.02% bromophenol blue, 20% glycerol, and 4% 2-mercaptoethanol, and then were heated at 95°C for 5 min. The extracted protein was subjected to Western blotting. In brief, 50 μg aliquots of protein were size-fractionated in a single dimension by SDS-PAGE (6–10% gels) and transblotted to 0.45 μm polyvinylidine difluoride membranes (IPVH304F0, Millipore, Billerica, MA) with a semi-dry electroblotting apparatus (Bio-Rad, Richmond, CA).

The blots were then washed three times in TBS with 0.1% Tween-20 (TBST) and incubated for 1 hour at room temperature in blocking buffer (Block Ace, Dainipponseiyaku, Osaka, Japan). Subsequently, the blots were incubated with an appropriate primary antibody for 1 h at room temperature or overnight at 4°C. Excess antibody was removed by washing the membrane with TBST three times for 10 min each. Then the membrane was incubated with a horseradish peroxidase-conjugated secondary antibody for 1 h at room temperature, followed by an addition of TBST. Reaction products were detected with the enhanced chemiluminescence system (Amersham, Buckinghamshire, United Kingdom). The membranes were treated with chemiluminescence reagents according to the manufacturer's protocol, and were exposed to X-ray films for 5–120 sec.

### Dual luciferase assay

We prepared the midkne 0.6-luc vector, in which the 609-base pair genomic DNA fragment of the midkne gene was cloned into the pGL2-basic vector (Promega, Madison, WI) and the firefly luciferase gene was included without a promoter sequence[24].

The transcripitional activity of a number of pancreatic cancer cell lines was measured with this dual luciferase reporter assay system (Promega, Madison, WI). Midkine 0.6-luc and a control vector (the renilla luciferase gene fused with the HSV-TK promoter (pRL-TK, Promega, Madison, WI) at a molar ratio of 10:1) were transfected together into target cells using Lipofectamine 2000 (Invitrogen, Carlsbad, CA). The cells were lysed after 2 days and luciferase activity was measured according to the manufacturer's protocol. The relative firefly luciferase activity of each cell lysate was calculated from the level of luminescence.

### Adenoviruses and adenoviral transduction analysis

We prepared recombinant adenovirus type 5 containing the 0.6 kb midkne promoter (Ad5MK) for midkne-regulated expression of E1A[24]. Type 5, E1A-deleted, replication-defective adenovirus containing the green fluorescent protein gene (Ad5GFP) was constructed using AdEasy XL Adenoviral Vector System (Stratagene, La Jolla, CA) according to the manufacturer's protocol. Adenoviruses were propagated in HEK 293 cells, purified by two rounds of cesium chloride density centrifugation, dialyzed, and stored at -70°C. Viral titers were determined with an Adeno-X Rapid Titer Kit (BD Biosciences Clontech, Palo Alto, CA).

To assess the efficiency of adenoviral transduction in human pancreatic cancer cells, we performed fluorescent staining using Ad5GFP. Pancreatic cancer cells were seeded onto coverslips and infected with at recombinant adenovirus at various multiplicities of infection (MOIs). After 48 hours, coverslips were mounted on the glass slides with Vectashield mounting medium (Vector Labolatories, Burlingame, CA), and the cells were examined under a fluorescence microscope (Olympus, Tokyo, Japan).

### Assessment of adenoviral replication

First, cells were infected with Ad5MK at various MOIs for 1 h and then the virus was removed. The infected cells were lysed in RIPA buffer to extract proteins after culture for 48 h. The proteins were subjected to SDS-PAGE and expression of E1A protein was analyzed by Western blotting. Next, cells were infected with Ad5MK at 1 MOI for 1 h and the medium was then refreshed. After the cells were cultured for 2 days, the cell lysate was prepared with three cycles of freezing and thawing.

HEK293 cells were infected with serially diluted cell lysates or tissue lysates. After 48 hr, the cells were stained with anti-adenoviral hexon protein antibody by using an Adeno-X rapid titer kit (BD Biosciences Clontech, Palo Alto, CA).

### *In vitro *cytotoxicity test

Pancreatic cancer cells were plated into 12-well plates in triplicate at a density of 1.0 × 10^4 ^cells/well. After 24- to 36 h of culture, cells were infected with Ad5GFP or Ad5MK at various MOIs for 1 h, and the infecting medium was replaced with complete medium. After 1, 3 and 5 days, the number of viable cells was counted using a cell counter (Coulter Z1, Beckman-Coulter, Fullerton, CA).

### Animal study

The animal study was performed in accordance with the guidelines for animal experiments of the Institute of Laboratory Animals at Kyoto University. Six-week-old male BALB/c nude mice were purchased from CLEA Japan (Tokyo, Japan). First, the mice were subcutaneously inoculated with Suit-2 cells (2 × 10^6^/ml) in 100 μl of Hank's balanced salt solution (HBSS) (Gibco-BRL) containing 20% matrigel (BD Biosciences, Bedford, MA). When the tumors reached about 10 mm in diameter, Ad5GFP or Ad5MK (2 × 10^9 ^PFU, 0.1 ml/mouse) was injected intratumorally. The mice were sacrificed at 3 or 7 days after adenoviral injection to extract RNA and lysates from the tumors. RT-PCR analysis of human adenovirus type 5 E1A and staining with anti-adenoviral hexon antibody were performed to assess the replication of adenoviruses *in vivo*.

Next, Suit-2 cells (2 × 10^6^/ml) in 500 μl of sterile PBS were inoculated into the peritoneal cavity of BALB/c nude mice to create a peritoneal dissemination xenograft model. The mice were divided into the following 4 groups: (1) an Ad5MK group, (2) an Ad5GFP group, (3) a PBS group, and (4) an untreated group. Ad5MK (2 × 10^9 ^PFU, 0.5 ml/mouse), Ad5GFP (2 × 10^9 ^PFU, 0.5 ml/mouse) or PBS (0.5 ml/mouse) was administered intraperitoneally at 4 days after the injection of Suit-2 cells. Survival was measured from the start of treatment.

### Statistical analysis

Quantitative data are presented as the mean ± SEM. Each *in vitro *experiment was performed independently at least three times. To compare mRNA levels in pancreatic tissue samples, Wilcoxon's rank sum test was used. Survival rates were calculated by the Kaplan-Meier method, and differences between groups were evaluated with the log-rank test and Wilcoxon's test. Statistical analysis was done by using JMP statistical software and statistical significance was considered to be present at p < 0.05.

## Results

### Midkine expression by human pancreatic cancer cell lines

We examined the expression of midkine mRNA in seven human pancreatic cancer cell lines by TaqMan PCR (Table 1). Midkine mRNA expression was strong in AsPC-1 and CFPAC-1 cells, but it was weak in MIAPaCa-2 cells.

**Table 1:** Expression of midkine mRNA in human pancreatic cancer cells.

Cell line	Midkine mRNA/β-actin mRNA
AsPC-1	1.19 ± 0.04
BxPC-3	0.37 ± 0.01
CFPAC-1	1.42 ± 0.02
HPAC	0.31 ± 0.01
MIAPaCa-2	0.001 ± 0.0004
PANC-1	0.02 ± 0.001
Suit-2	0.13 ± 0.003

Data are expressed as the mean ± SEM.

Next, midkine protein expression was assessed by Western blot analysis (Figure 1A). AsPC-1 and CFPAC-1 cells showed strong expression of midkine protein, whereas BxPC-3, HPAC and Suit-2 cells showed moderate expression. In contrast, expression by PANC-1 cells was weak and MIAPaCa-2 cells showed no midkine band. The extent of midkine protein expression was in parallel to that of midkine mRNA expression. In the following experiments, we therefore designated the MIAPaCa-2 cell line as midkine-negative.

**Figure 1:** **Midkine protein expression by human pancreatic cancer cell lines and human pancreatic cancer tissues**. (A) Midkine protein expression by human pancreatic cancer cell lines. AsPC-1 and CFPAC-1 cells showed strong expression of midkine protein, whereas BxPC-3, HPAC, and Suit-2 cells showed moderate expression. In contrast, expression by PANC-1 cells was low and MIAPaCa-2 cells showed no detectable midkine band. (B) Midkine mRNA expression in non-cancerous pancreatic tissues and human pancreatic cancers. Expression of midkine mRNA in the pancreatic cancers was significantly stronger than in the non-cancerous pancreatic tissues (p < 0.001).

### Midkine expression in human pancreatic cancer

We assessed the expression of midkine mRNA in 22 pancreatic cancer samples and 18 adjacent non-cancerous pancreatic tissue samples by TaqMan PCR (Figure 1B). The midkine mRNA/β-actin mRNA ratio of pancreatic cancer and non-cancerous pancreatic tissue was 0.60 ± 0.55 and 0.22 ± 0.13, respectively. Expression of midkine mRNA was significantly stronger in pancreatic cancer than in non-cancerous tissue (p < 0.001).

### Transcriptional activity of the midkine promoter in human pancreatic cancer cells

We investigated the transcriptional activity of the midkine promoter by the dual luciferase reporter assay in AsPC-1, CFPAC-1, MIAPaCa-2, PANC-1, and Suit-2 cells (Table 2). This assay showed that the relative luciferase activity mediated by the 0.6 kb midkne fragment in AsPC-1, PANC-1, and Suit-2 cells was approximately 6 to 20 times greater than that in midkne-negative MIAPaCa-2 cells. Transcriptional activity in MIAPaCa-2 cells was extremly low. The transcriptional activity in each of the cell lines was usually correlated with the expression of midkne, although CFPAC-1 cells showed low transcriptional activity and high midkne expression.

**Table 2:** Transcriptional activity of MK promoter in human pancreatic cancer cells.

Cell lines	Relative luciferase activity
AsPC-1	0.57 ± 0.09
CFPAC-1	0.06 ± 0.01
MIAPaCa-2	0.03 ± 0.01
PANC-1	0.16 ± 0.02
Suit-2	0.29 ± 0.01

Relative luciferase activity was defined as firefly luciferase activity per renilla luciferase activity in cancer cells. Data are expressed as the mean ± SEM.

### Sensitivity of human pancreatic cancer cell lines to adenovirus infection

We examined the induction of Ad5GFP in human pancreatic cancer cells (Figure 2). Cells were infected with Ad5GFP (1, 10, or 25 MOI) at 16 to 18 h after seeding. After 48 h, GFP-expressing cells were detected by fluorescence microscopy. We found that pancreatic cancer cells exhibited a heterogeneous adenoviral transduction profile. Many of the CFPAC-1 and Suit-2 cells infected at an MOI of 25 expressed GFP, whereas AsPC-1 cells showed far lower adenoviral transduction efficiency. We also found that the number of GFP-expressing cells increased in an MOI-dependent manner.

**Figure 2:** **Sensitivity of human pancreatic cancer cell lines to adenovirus infection**. Pancreatic cancer cells were infected with Ad5GFP (1, 10 or 25 MOI) at 16 to 18 h after seeding. After 48 h, GFP-expressing cells were detected by fluorescence microscopy. (Original magnification ×100).

### Ad5MK shows specific replication and infectivity for human pancreatic cancer cell lines

Since the adenoviral infection cycle is completed within 24 h, E1A expression by infected cells after 48 h reflects viral replication. Therefore, to determine the specificity of Ad5MK replication, we used pancreatic cancer cell lines with different levels of midkine expression and then examined E1A expression by Western blotting (Figure 3A). We found that viral replication was dependent on the MOI of infection.

**Figure 3:** **Replication specificity and infectivity of Ad5MK for human pancreatic cancer cell lines**. (A) E1A protein expression by pancreatic cancer cells. Pancreatic cancer cell lines were infected with Ad5MK showing different levels of midkine expression, Ad5GFP alone, or the vehicle. (B) Adenoviral hexon staining. HEK293 cells were treated with preparations of Ad5MK-infected pancreatic cancer cells. After 48 hr, HEK293 cells were stained with anti-adenoviral hexon antibody. (Original magnification ×100)

Next, we examined the infectivity of Ad5MK prepared from pancreatic cell line in HEK293 cells by using an anti-adenoviral hexon antibody (Figure 3B). Stained HEK293 cells were found after infection with preparations from midkine-positive cells (PANC-1, Suit-2, AsPC-1, and CFPAC-1), whereas there were no stained cells after infection with a preparation from midkine-negative MIAPaCa-2 cells.

### Specific cell killing effect of Ad5MK *in vitro*

We subsequently examined the ability of Ad5MK to kill pancreatic cancer cells (Figure 4). The number of viable cells was counted by using a Coulter counter. Ad5MK showed a much stronger-killing effect against Suit-2 and PANC-1 cells that have moderate and weak midkine expression, respectively, compared with its effect on midkine-negative MIAPaCa-2 cells.

**Figure 4:** ***In vitro *cytotoxicity of Ad5MK**. Pancreatic cancer cells were plated in triplicate in 12-well plates at 1.0 × 10^4 ^cells/well. After 24 to 36 h, the cells were infected with Ad5GFP or Ad5MK at various MOIs. After 1, 3, and 5 days, the number of viable cells was counted.

On the other hand, moderate cell-killing effect against CFPAC-1 cells was found in 10 MOI of Ad5MK. CFPAC-1 cells had high midkine expression and moderate efficiency of adenoviral transduction. Transcriptional activity of midkine promoter in CFPAC-1 cells was low, but it was higher compared to that of MIAPaCa-2 cells. This may be the reason why growth suppression of CFPAC-1 cells was observed by 10 MOI of Ad5MK. In contrast, Ad5MK had no effect on AsPC-1 cells as far as the designated conditions, although these cells showed strong midkine expression. This finding may have reflected low efficiency of adenoviral transduction. Ad5GFP had no influence on the growth of any of the cells in this assay compared with normal control cells (data not shown).

### Adenoviral replication and anti-tumor effect of Ad5MK *in vivo*

We assessed adenoviral replication *in vivo *by using a Suit-2 subcutaneous xenograft model of pancreatic cancer. RNA and tumor lysates were obtained from the subcutaneous xenografts after injection of adenoviruses. RT-PCR analysis for human adenovirus type 5 E1A showed that E1A expression could be detected in the Ad5MK groups (Figure 5A). On the other hand, no band was seen in the untreated and Ad5GFP groups. After staining with anti-adenoviral hexon antibody, positive cells were only found in the Ad5MK groups, whereas there were no positive cells in the untreated and Ad5GFP groups (Figure 5B).

**Figure 5:** **Replication of adenovirus in a Suit-2 subcutaneous xenograft model of pancreatic cancer**.(A) Human adenovirus type 5 E1A expression. RNA was extracted from subcutaneous tumors after injection of adenoviruses. Expression of E1A was analyzed by RT-PCR. (B) Adenoviral hexon staining. HEK293 cells were infected with Ad5MK prepared from subcutaneous xenografts after injection of adenoviruses. After 48 hr, HEK293 cells were stained with anti-adenoviral hexon antibody. Positive cells were only found in the Ad5MK groups, whereas there were no positive cells in the untreated and Ad5GFP groups. (Original magnification ×100)

Finally, we assessed the anti-tumor effect in a Suit-2 intraperitoneal xenograft model after the intraperitoneal injection of Ad5MK (Figure 6). Following the inoculation of 2 × 10^6^/ml Suit-2 cells into the peritoneal cavity of nude mice, 2 × 10^9 ^PFU of Ad5MK or Ad5GFP, or 500 μl of PBS, was administered intraperitoneally. In this intraperitoneal xenograft model, our preliminary study revealed that untreated mice died of peritoneal dissemination with bloody ascites after approximately 2 to 3 weeks. Almost all of the mice in the untreated, PBS, and Ad5GFP groups died within 35 days, whereas almost all of the mice in the Ad5MK group survived for more than 50 days. There was a statistically significant difference of the survival time between the Ad5MK group and the other group.

**Figure 6:** **Anti-tumor effect of Ad5MK in a Suit-2 intraperitoneal xenograft model**. After intraperitoneal inoculation of 2 × 10^6^/ml Suit-2 cells in nude mice, 2 × 10^9 ^PFU of Ad5GFP or Ad5MK, or 500 μl of PBS, was administered intraperitoneally. There was a significant difference of survival time between the Ad5MK group and the other groups (p = 0.0002 Log-rank test and p = 0.0002 by Wilcoxson's test).

## Discussion

Conditionally replicative adenoviruses, which show tumor-specific replication and oncolysis, are a promising new treatment modality for malignancies resistant to conventional therapies [25,26]. In this study, we demonstrated a possible strategy for pancreatic cancer based on Ad5MK replication-competent adenovirus. Midkine expression is increased in various human tumors, including gastrointestinal cancers [19-22]. We showed that most human pancreatic cancer cell lines (6 out of 7 lines tested) express midkine to some extent and that the level of midkine mRNA expression in pancreatic cancer tissues is significantly higher than in non-cancerous pancreatic tissues. These findings suggested that the midkine promoter may be a potential candidate for safe suicide gene therapy targeting pancreatic cancer.

We next examined the promoter activity of midkine in a dual luciferase reporter assay. A 2.3-kb fragment from the 5' region of the midkine gene contains the elements responsible for promoter activity [27]. Within this 2.3-kb fragment, Yoshida et al. have demonstrated the presence of a cis-element with strong promoter activity located at the -559/50 region using the CAT assay, and they also reported that its midkine promoter activity in tumor cells was comparable to that of the SV40 early promoter [28]. Therefore, we examined the promoter activity of this 0.6-kb fragment in human pancreatic cancer cells by using the dual luciferase reporter assay. We showed that the relative luciferase activity in AsPC-1, PANC-1, and Suit-2 cells was greater than that in midkne-negative MIAPaCa-2 cells. Transcriptional activity in the cell lines was generally parallel to the level of midkne expression. In CFPAC-1 cells, however, the level of midkne expression did not correspond well with the transcripitional activity of the midkne promoter. We cannot explain this discrepancy, but it has been reported that the level of endogenous midkne expression and its promoter activity are not always correlated with each other because of various factors such as negative and positive regulatory elements residing outside the region analysed [29]. Another possible explanation may be differences between cell lines with respect to regulation of the proteins involved in transcription [29].

Because the efficiency of adenoviral transfection varies between cell lines, it was essential to examine the infectivity of Ad5GFP for multiple human pancreatic cancer cell lines. Adenoviral transduction efficiency was far lower for AsPC-1 than the other cell lines. Adenoviral replication in AsPC-1 cells was lower than in any other midkine-positive cell line and no killing of AsPC-1 cells was observed at 10 MOI, although these cells showed high midkine expression and transcriptional activity. Thus, we consider that adenoviral transduction efficiency as well as transcriptional activity is critical for adenovirus-mediated gene therapy. In pancreatic cancer cells, the combined efficiency of transduction and transcription determines the actual cell-killing effect of Ad5MK.

When clinical application is considered, not only anti-tumor activity but also toxicity for normal tissues should be taken into account. In this regard, Ad5MK showed specific cytotoxicity for midkine-positive cells both *in vitro *and *in vivo*. Despite the target selectivity of Ad5MK, weak E1A expression was found in midkine-negative cells after infection with 5 MOI of Ad5MK. Type 5 adenoviruses are commonly used in viral therapy experiments, but show species-specific replication, and it has been reported that these adenoviruses do not replicate in mice or rats. There are no suitable animal models apart from the cotton rat to assess the toxicity of conditionally replicative adenoviruses, but replicative viruses have already shown at least low-level viral production and/or systemic toxicity in clinical trials[25,30,31]. The precise requirements for selective targeting to prevent damage to normal tissues *in vivo *need to be clarified in the future.

We demonstrated an anti-tumor effect of Ad5MK on midkine-positive tumor cells *in vivo *as well as *in vitro*. Our animal studies showed that mice treated with Ad5MK survived for significantly longer than the other groups. Even in the Ad5MK group, however, half of the mice died due to peritoneal dissemination after about 50 days. This may have been due to an inadequate dose of adenovirus or because of the regrowth of cancer cells with resistance to adenovirus-mediated gene therapy. In this study, we only gave a single dose of adenovirus intraperitoneally after tumor cell inoculation. In the future, we should investigate the optimum volume and number of adenovirus doses to improve the efficacy of Ad5MK treatment. Another way to improve the results could be employment of fiber-modified adenoviruses, which can enter cancer cells resistant to conventional adenoviral gene transfer in a coxsackievirus and adenovirus receptor (CAR)-independent manner.

## Conclusion

Midkine expression was increased in pancreatic cancer cell lines and pancreatic cancer tissues. Ad5MK showed specific targeting of and cytotoxicity for midkine-positive cells both *in vitro *and *in vivo*. These results suggest that replication-competent adenoviruses based on the midkine promoter might have the potential to be used in gene therapy for pancreatic cancer.

## Competing interests

The authors declare that they have no competing interests.

## Authors' contributions

ET conceived of the study and performed experiments on adenoviruses. RD conceived of the study, and participated in its design and coordination and helped to draft the manuscript. KK conceived of the study and performed experiments on mice. TM conceived of the study and performed experiments on mice. DI conceived of the study and performed experiments on pancreatic cancer cell lines. MK conceived of the study and performed experiments on pancreatic cancer cell lines. AK conceived of the study and performed experiments on pancreatic cancer cell lines. KN conceived of the study and performed experiments on mice. TI conceived of the study and performed experiments on mice. TM conceived of the study and performed experiments on pancreatic cancer cell lines. MW conceived of the study, and participated in its design and coordination and helped to draft the manuscript. MT conceived of the study, and participated in its design and coordination and helped to draft the manuscript. SU conceived of the study, and participated in its design.
